The article "Inflation Prediction Method Based on Deep Learning" was published in 2021. Journal: Comput Intell Neurosci.

# Inflation Prediction Method Based on Deep Learning

**DOI:** 10.1155/2021/1071145

**Published:** 2021-08-19

**Authors:** Cheng Yang, Shuhua Guo

**Affiliations:** School of Economics, Yunnan University, Kunming 650000, China

## Abstract

Forward-looking forecasting of the inflation rate could help the central bank and other government departments to better use monetary policy to stabilize prices and prevent the impact of inflation on market entities, especially for low- and middle-income groups. It can also help financial institutions and investors better make investment decisions. In this sense, the forecast of inflation rate is of great significance. The existing literature mainly uses linear models such as autoregressive (AR) and vector autoregressive (VAR) models to predict the inflation rate. The nonlinear relationship between variables and the mining of historical data information are relatively lacking. Therefore, the prediction strategies and accuracy of the existing literature need to be improved. The predictive model designed in deep learning can fully mine the nonlinear relationship between variables and process complex long-term time series dynamic information, thereby making up for the deficiencies of existing research. Therefore, this paper employs the recurrent neural networks with gated recurrent unit (GRU-RNN) model to train and analyze the Consumer Price Index (CPI) indicators to obtain inflation-related prediction results. The experimental results on historical data show that the GRU-RNN model has good performance in predicting China's inflation rate. In comparison, the performance of the proposed method is significantly better than some traditional models, showing its superior effectiveness.

## 1. Introduction

The inflation rate is one of the important indicators for monitoring the operation of the macroeconomy. So, it is of great significance to make forward-looking forecasts of the inflation rate for the adjustment of the policies [1–4]. First, one of the important goals of monetary policy is to stabilize prices. However, there is a certain time lag in the process of monetary policy regulating prices. Therefore, the central bank needs more accurate inflation forecasts as a prerequisite to better use monetary policy to stabilize prices. Second, the inflation rate not only affects investors' decisions in the investment cycle but also affects investors' decisions in investment products. Therefore, it is of great guiding significance for the financial institutions and investors to predict the inflation rate. Third, the existence of large family property gaps and frequent structural inflation has made inflation more harmful to low- and middle-income groups, thus further highlighting the necessity and importance of predicting the inflation rate. In current China, the property of the low- and middle-income class mainly exists in the form of deposits, while the property of the high-income class exists in the form of real estate, etc. Inflation will reduce the real interest rate and cause the savings of low- and middle-income families to shrink, while high-income families may benefit from rising housing prices. In addition, the structural inflation characterized by sharp increases in food prices often occurs in China, and the proportion of food expenditures in the middle- and low-income groups is relatively high. The existence of these two phenomena makes it difficult for low- and middle-income groups to withstand the impact of inflation. Even moderate inflation will have a more serious adverse effect on low- and middle-income groups. Therefore, the precise forecast of the inflation rate has great influences on the country's policies and citizens' daily lives.

The article "Inflation Prediction Method Based on Deep Learning" was published in 2021. Journal: Comput Intell Neurosci.

In terms of the prediction of the Consumer Price Index (CPI), the relevant literature mainly uses five types of models to conduct research. The first one is the Phillips curve model, and related research can be found in [5–7]. The second is time series models such as autoregressive (AR), autoregressive moving average (ARMA), and autoregressive integrated moving average (ARIMA), and the relevant works can be found in [8–10]. The third is the vector AR (VAR), structural AVR (SVAR), and Bayesian VAR (BVAR) series models with some medications to the second type of models. Some related researches are reported in [11–14]. The fourth is the term structure model of interest rates with some representative works in [15]. The fifth uses neural network models such as back propagation (BP), and related researches are reflected in [16–22]. Specifically, when predicting the inflation rate, existing studies mainly focus on linear models, and there are relatively few studies on nonlinear models. In contrast, in the past ten years, some literatures have gradually strengthened the use of nonlinear machine learning methods represented by neural networks when predicting gross domestic product (GDP), and the types of data that can be processed are more complex, including nonlinear, high-frequency, and higher-dimensional ones. Based on the results of these literatures, the nonlinear model represented by neural network performs better than traditional linear models such as AR or ARMA in predicting the inflation rate. This is because the impact of monetary policy and many other factors on the inflation rate is likely to be nonlinear, which largely determines that the prediction precision of the nonlinear model is better than the linear model. We take the effect of quantitative monetary policy on interest rates as an example. There are many effects including the liquidity, income, price, and inflation expectation and it may occur that some effects are opposite to the others. Therefore, the quantity monetary policy affects the interest rate and then has a complex and even nonlinear impact on aggregate demand and inflation.

The article "Inflation Prediction Method Based on Deep Learning" was published in 2021. Journal: Comput Intell Neurosci.

Although traditional neural network models such as BP can identify the nonlinear relationship between variables, they cannot reflect the time series relationship between variables. In the economic field, the temporal relationship between variables and the logical relationship behind them are very important. In recent years, the deep learning theory developed fast with a rich set of tools, which has been widely used in signal, image processing, data mining, etc. Also, the deep learning models have excellent time series data processing capabilities, which achieved good results in the field of economic and financial forecasting [23–27]. Among them, the recurrent neural network (RNN) model is based on the ordinary multilayer BP neural network, adding the horizontal connection between the units of the hidden layers. Through a weight matrix, the value of the previous time series neuron can be transferred to the current neuron so that the neural network has the memory. The gated RNN (GRU-RNN) [28–31] is an improved form of RNN. By introducing different “gating” mechanisms in the hidden layer nodes of the RNN, it can process long-interval time series signals to get more data characteristics and time dependence. Owing to the merits and advantages of GRU-RNN, this paper introduces it into inflation forecasting. Using historical economic data as input, the designed GRU-RNN is trained to obtain an end-to-end prediction network. In the application process, the current relevant economic indicators are used as input to obtain the predicted value of the inflation-characterized quantity. In the experiment, the proposed method was tested and compared with several types of existing models based on China's historical CPI data. The results reflect the effectiveness of the proposed method.

## 2. Basics of GRU-RNN

GRU-RNN is an improved form of RNN, which could achieve higher precision and robustness [28–31]. In a simple way for explanation of RNN, some outputs of its neuron can be used as its input to be transmitted to the neuron again, and historical information can be retained and used, which is very effective for dealing with timing problems.

As shown in Figure 1, the architecture of RNN is composed of an input layer **X**, a hidden layer **H**, and an output layer **Y**. Compared with the conventional neural networks, RNN has an extra delayer that retains historical information. W, U, V are the input layer, output layer, and weight matrix of the hidden layer from the previous moment to the current hidden layer, respectively. Afterwards, at the time moment of *t*, the state of the hidden layer *h*_*t*_ is determined by the current input x_*t*_ and the state of the previous hidden layer h_*t*−1_ jointly, which is described as follows:

(1) $$\begin{array}{c} h_{t}=\varphi \left({\text{Uh}}_{t-1}+{\text{Wx}}_{t}+b\right), \end{array}$$

(2) $$\begin{array}{c} y_{t}={\text{Vh}}_{t}, \end{array}$$

where *φ*(•) is the nonlinear active function; *b* is the bias.

The article "Inflation Prediction Method Based on Deep Learning" was published in 2021. Journal: Comput Intell Neurosci.

Although RNN has achieved good results in solving many timing prediction problems, the long-term sequences and complex hidden layers may cause gradients to explode or disappear in the process of error back propagation. In order to solve the problem of long-term dependence of RNN, while reducing the requirements for computational overhead and storage space and increasing the convergence speed, GRU-RNN was proposed. GRU-RNN mainly introduces the network door mechanism to control the path of information transmission. Among them, the update gate determines the degree of influence of the state at the previous moment on the state at the current moment, and the reset gate determines the degree of combination between the current input and the state at the previous moment.  Figure 2 shows the structure of the hidden layer node in GRU-RNN.

As shown in Figure 2, it can be concluded that the calculation for GRU-RNN to obtain the output of hidden layer *h*_*t*_ is as follows:

(3) $$\begin{array}{c} z_{t}=\sigma \left(w_{z}\cdot \left[h_{t-1},x_{t}\right]+b_{z}\right),\\ f_{t}=\sigma \left(w_{r}\cdot \left[h_{t-1},x_{t}\right]+b_{r}\right),\\ {\tilde{h}}_{t}=\tan\;h\left(w_{\tilde{h}}\cdot \left[f_{t}⊙h_{t-1},x_{t}\right]+b_{\tilde{h}}\right),\\ h_{t}=\left(1-z_{t}\right)⊙\;h_{t-1}+z_{t}⊙{\tilde{h}}_{t}, \end{array}$$

where *x*_*t*_, *h*_*t*−1_, *z*_*t*_, and *f*_*t*_ are the input, output, update gate output, and reset gate output of the GRU-RNN hidden layer node, respectively. The input *x*_*t*_ and the previous hidden layer output *h*_*t*−1_ jointly determine the amount of process ${\tilde{h}}_{t}$; *w* and *b* are the weight parameters and bias parameters obtained from training; ⊙ represents the multiplication of corresponding position elements in the matrix; *σ* and tanh represent the sigmoid function and the hyperbolic tangent function, respectively. Based on the above solution, the output, i.e., the precited value, can be obtained from equation (2).

The article "Inflation Prediction Method Based on Deep Learning" was published in 2021. Journal: Comput Intell Neurosci.

Figure 3 shows the main process of inflation prediction based on GRU-RNN, which can be summarized as the following steps:

  Step 1: The acquisition of the training data: the feature vectors are constructed to describe inflation as the inputs for training GRU-RNN, and the corresponding inflation indicators are used as the outputs.
  Step 2: The establishment of a GRU-RNN with preset network parameters: the network structure is constructed and the appropriate activation function, objective function, optimization algorithm, and evaluation function are selected. The convolutional neural network sampling interval, number of training iterations, learning rate, and other hyperparameters are set. The network weights and biases are initialized.
  Step 3: Train of the GRU-RNN: the optimization algorithm is used to realize the learning of parameters such as network weights and offsets until the objective function meets the requirements. Finally, the optimal parameters of the networks can be found.
  Step 4: Estimation of the inflation indicator: the newly collected inflation feature vector is input into the trained network and the estimated value of inflation indicator is output.

Based on the above steps, the economic data can be analyzed to find its inner relationship with the help of GRU-RNN. There are two issues that should be considered. The first one is how to design and construct the feature vector to describe the inflation. Actually, there are many economic indexes related to the inflation. A concise and effective one should be developed to enhance both the efficiency and precision of the prediction of the inflation. In this paper, we choose several closely related economic indexes to construct the feature vector, which will be detaily explained in the experiments. The second one is how to select the indicator for the inflation. Similar to the first case, a representative parameter should be used to truly reflect the condition of the inflation. In this paper, we use the CPI as the indicator of the inflation.

## 3. Experiments and Analysis

### 3.1. Dataset and Evaluation Index

#### 3.1.1. Introduction of the Used Data

All the relevant samples used in this paper are monthly data, and the relevant data come from the China economic website and Wind database. Among them, the Shanghai and Shenzhen 300 index (STOCK), the 7-day interbank offered rate (RATEST), the central parity of the RMB against the US dollar (EXC), and the wheat futures closing price index (CBOT) can directly query daily data. We take the average of each day's data contained in each month of these indicators to obtain monthly data. For the remaining indicators, monthly data can be directly obtained. Based on the availability of data, when predicting CPI, the beginning and ending time of the sample selected in this article is from April 2005 to June 2021, and contains a total of 195 sample observations. These samples will be used as the training samples to train the designed GRU-RNN and also used as the references to calculate the errors for prediction.

The article "Inflation Prediction Method Based on Deep Learning" was published in 2021. Journal: Comput Intell Neurosci.

#### 3.1.2. Construction of Features

According to the existing literature, this paper constructs a benchmark feature vector to describe the inflation including 11 variables: CPI year-on-year growth rate (CPI), which measures inflation rate, is one of the key indicators to be predicted in this paper; the year-on-year growth rate (M1) of the narrow money supply, the year-on-year growth rate of the broad money supply (M2), and the 7-day interbank lending rate (RATEST) reflect the impact of quantitative monetary policy and price-based monetary policy on the inflation rate, respectively; industrial increase of the year-on-year growth rate (IVA) is used to reflect the impact of the activity of production activities on the inflation rate; the year-on-year growth rate of total retail sales of consumer goods (C) is used to reflect the impact of consumer demand on the inflation rate; the national housing boom index (HINDEX), the cumulative year-on-year growth rate of real estate development investment (HINVEST), and the year-on-year growth rate of newly started area of commercial housing this year (HSTARTS) are used to fully reflect the impact of the operation of the real estate market on the inflation rate; the Shanghai and Shenzhen 300 index (STOCK) is used to reflect the impact of the stock market on the inflation rate; the central parity of the RMB against the US dollar (EXC) is used to reflect the impact of changes in the exchange rate market on the inflation rate. These 11 variables jointly construct a feature vector to describe the CPI, which is used as the input of GRU-RNN to train the network.

#### 3.1.3. Evaluation Index

When judging the predictive performance of different models, some quantitative evaluation indexes are necessary. According to the existing literature [3, 8, 12], this paper chooses three indicators of mean squared error (MSE), mean absolute percent error (MAPE), and symmetric mean absolute percentage error (SMAPE) as the indexes for the evaluation of the prediction performance of CPI. The three indexes are defined as follows:

(4) $$\begin{array}{c} \text{MSE}=\frac{1}{N}\sum_{\tau =t_{0}}^{t_{N-1}}{\left(y_{\tau }-y_{\tau }^{0}\right)}^{2}a,\\ \text{MAPE}=\frac{100\%}{N}\sum_{\tau =t_{0}}^{t_{N-1}}\left|\frac{y_{t}-y_{t}^{0}}{y_{t}^{0}}\right|,\\ \text{SMAPE}=\frac{100\%}{N}\sum_{\tau =t_{0}}^{t_{N-1}}\frac{\left|y_{t}-y_{t}^{0}\right|}{\left(\left|y_{t}\right|+\left|y_{t}^{0}\right|\right)/2}, \end{array}$$

The article "Inflation Prediction Method Based on Deep Learning" was published in 2021. Journal: Comput Intell Neurosci.

## 4. Results and Analysis

Based on real historical data, the three evaluation indexes of MSE, MAPE, and SMAPE are used to test and analyze the proposed method and several types of comparison methods. The statistics of the results are shown in Table 1. It can be seen that the index values of MSE, MAPE, and SMAPE predicted by the GRU-RNN method in this paper are all less than the corresponding index values obtained by the comparison methods, indicating that the GRU-RNN model is more suitable for CPI prediction than the others. Taking the MSE index as an example, the performance of the GRU-RNN and BP methods is better than those achieved by the ARMA and BVAR methods, showing the significant advantages of neural networks in data prediction. Comparing the two networks of GRU-RNN and BP, the former has a further smaller MSE value, indicating that its prediction accuracy has been further improved. As a shallow-layer neural network, BP has limited capabilities in nonlinear data processing and has certain shortcomings for more complex CPI predictions. With a deep network structure, RNN has significantly enhanced nonlinear data acquisition capabilities and has stronger processing capabilities for CPI prediction. As an improved form of RNN, GRU-RNN not only inherits the advantages of RNN in data prediction but also further improves the prediction accuracy through the introduction of gate nodes. The indicator trends of MAPE and SMAPE are basically the same as MSE, and both can reflect the significant advantages of GRU-RNN in CPI prediction.

Furthermore, this paper adds a certain degree of random noise to historical data. Specifically, a certain degree of uncertainty is added to each of the 11 elements in the feature vector, and the degree of deviation is set to 2%, 4%, 6%, and 8%, respectively. Under this condition, the final prediction accuracy of various methods has been reduced to a certain extent.  Table 2 takes the MSE index as an example and lists the results of different methods at different noise levels. It can be seen that the proposed method can maintain the minimum MSE under each noise level, which proves the robustness of its prediction. In particular, under the condition that the noise interference becomes more and more serious, the advantages of the proposed method are more significant, which further demonstrates its effectiveness for the uncertain data.

## 5. Conclusion

This paper proposes a method based on GRU-RNN for inflation forecasting. As an improved version of RNN, GRU-RNN has certain advantages in sequence prediction performance. In the implementation of the proposed method, this paper uses CPI as the indicator of inflation and uses multiple economic-related indexes as the feature vector of CPI. With the historical data as input, the designed GRU-RNN is trained to optimize the network parameters. In the practical applications, the currently collected CPI feature vector is used as input to obtain the predicted value of CPI. In the experiments, historical actual data are used to test and analyze the performance of the method. Through comprehensive research and judgment of multiple evaluation indexes, the performance of the proposed method is better than several types of traditional models, which verifies its influence in inflation forecasting. The future works can be proceeded from two aspects. First, more effective feature vectors describing the inflation or CPI can be designed to train the networks, so the prediction precision can better reflect the real situation. Second, more suitable deep learning models with better prediction performance can be employed and improved for the application of predicting inflation.

The article "Inflation Prediction Method Based on Deep Learning" was published in 2021. Journal: Comput Intell Neurosci.

## Figures and Tables

**Figure 1:** Architecture of RNN unfolded in time.

**Figure 2:** Structure of the hidden layer node in GRU-RNN.

**Figure 3:** Illustration of the process of inflation prediction based on GRU-RNN.

**Table 1:** Comparison of different methods in the prediction of CPI.

Method	Evaluation index		
	MSE	MAPE	SMAPE
Proposed	0.359	0.460%	0.458%
ARMA	0.482	0.672%	0.683%
BVAR	0.421	0.602%	0.598%
BP	0.382	0.513	0.508

**Table 2:** Comparison of the MSE different methods in the prediction of CPI.

Method	Noise level			
	2%	4%	6%	8%
Proposed	0.372	0.432	0.503	0.594
ARMA	0.496	0.543	0.672	0.738
BVAR	0.453	0.514	0.624	0.722
BP	0.412	0.489	0.549	0.637

## Data Availability

The dataset used in this paper is publicly available.
